The article "The Application Value of CT Three-Dimensional Microscope Reconstruction Technology in the Diagnosis of Cervical Cancer" was retracted in 2023. Reasons: signs of a paper mill; compromised peer review; unreliable results or conclusions.

# The Application Value of CT Three-Dimensional Microscope Reconstruction Technology in the Diagnosis of Cervical Cancer

**DOI:** 10.1155/2022/5648195

**Published:** 2022-06-06

**Authors:** Shaoliang Sun, Xiye Wang, Yanjia Chen

**Affiliations:** ^1^Department of Radiology, Shengzhou People's Hospital, Zhejiang 312400, China; ^2^Department of Obstetrics and Gynecology, Shengzhou People's Hospital, Zhejiang 312400, China

## Abstract

In order to study the application value of CT three-dimensional microscope reconstruction technology in the diagnosis of cervical cancer. In this paper, 232 patients with newly diagnosed stage IA-II A2 and some stage III C: cervical cancer (stage IB1-IIA2 of stage f go in 2009) were selected, and 204 patients with stage IB1-IIA2 of stage 2009 fig 0 were selected. The original data of DICOM were obtained by CT scanning and imported into mics10.01 software to complete lymph node reconstruction. The short diameter value > 10 mm is used as the standard to judge whether the lymph node is metastatic. Referring to the 2018fig 0 staging standard, if it indicates that the lymph node is positive, it is IIICr stage. The gold standard is the diagnosis of III CP according to the surgical and pathological results, and then the diagnostic efficiency of III C stage is evaluated. The experimental results showed that 65 cases were diagnosed as IIIC stage, and 70 cases were diagnosed as IIICp stage. There was consistency between IIICr and IIICp stage, and the kappa value was 0.340. Using CT multiphase enhanced scanning and three-dimensional reconstruction technology to diagnose cervical cancer has high detection rate and high accuracy of staging diagnosis, which is worthy of clinical application.

## 1. Introduction

Every year, there are more than 490000 new cervical cancer patients worldwide, of which the number of new cervical cancer patients in China accounts for about 30% of the total number of patients in the world. In recent years, the society has been developing continuously, people's life rhythm is quickening, the pressure of women is increasing, and the degree of sexual openness is increasing, making the incidence rate of cervical cancer increasing year by year, and the group of patients is becoming younger. Studies have shown that since 2001, the incidence of cervical cancer in my country has increased by 13.5% every year, and the mortality rate has increased by 8.1% every year. Accurately diagnosing the stage of a patient's condition can improve treatment outcomes and reduce mortality. Traditional gynecological examinations are not very effective in diagnosing cervical cancer staging [1]. Spiral CT has high accuracy and short scanning time. After three-dimensional reconstruction, the images are more vivid and clear, and the diagnostic accuracy of various diseases is higher.

Imaging suggests that lymph node metastasis is classified as IIICr for these patients, 2021nccn guidelines do not recommend stratified treatment, and all recommend radiotherapy. Different scholars have different opinions [2]. Some scholars believe that direct surgical treatment can also be selected for young patients with lymph node metastasis (III CR) indicated by the imaging of go stage a-iia2 in 2009. On the one hand, the purpose of the operation is to evaluate and remove the pelvic and paraaortic lymph nodes more accurately, play a role in staging and reducing the tumor load, and avoid the damage of ovarian function caused by direct radiotherapy and chemotherapy. On the other hand, through postoperative pathology, we can understand whether there are high-risk factors affecting the prognosis of patients, such as lymph node metastasis and parauterine infiltration, so as to further determine whether radiotherapy and chemotherapy and radiotherapy irradiation field are needed for individualized treatment [3]. Of course, the difference in the prognostic effect between the two treatment regimens needs to be verified by further clinical prospective research data. Therefore, we should be cautious in the clinical diagnosis and treatment of stage III C. Considering that patients with positive lymph nodes need supplementary radiotherapy after operation, resulting in significantly increased total complications and decreased quality of life, it is very important for the treatment strategy decision and prognosis of patients with cervical cancer to further clarify the existence of lymph node metastasis through imaging before operation.

Imaging examination has important clinical significance in evaluating the accuracy of stage III C and studying the high-risk factors of lymph node metastasis. According to the clinical data of cervical cancer patients treated in O1, the application value of 3D reconstruction technology based on CT original data (Figure 1) in the MCR stage of cervical cancer was discussed, and the risk factors of cervical cancer lymph node metastasis were further analyzed. The second part of this study mainly constructs the digital three-dimensional model of in vivo lymph nodes through three-dimensional reconstruction technology, measures the short diameter and long diameter of their lymph nodes and calculates their ratio, discusses the value of different indicators to judge lymph node metastasis, and looks for a more suitable diagnostic standard for metastatic lymph nodes of cervical cancer [4].

## 2. Literature Review

Zhang et al. improved computed tomography (CT) equipment and improved image processing techniques, showing that CT can not only accurately reflect the morphological characteristics of primary cervical cancer and distant lymph node metastasis, but also reflect the pathophysiological characteristics of cervical cancer. [5]. Xiao et al. believed that the spectral CT imaging technology uses kV fast conversion technology to obtain monochromatic images of various energy units and weakens the iodine contrast through material separation technology, so that the iodine concentration can be calculated [6]. Li et al. expand the use of traditional CT scans to provide hospitals with more metrics and diagnostic tools. However, few studies have reported the application of spectral imaging in cervical cancer. The 640-line CT three-dimensional energy spectrum imaging can be completed in only two times [7]. Zhang and others found that sure exposure smart Ma technology can automatically match different kV, maintain consistent noise level, and obtain the best image quality [8]. Konarev and others believe that the combination of 3D adaptive iterative dose reduction (aidr-3d) reconstruction technology can effectively reduce the radiation dose of CT energy spectrum imaging of cervical cancer [9]. Zhang and Zhu believe that compared with conventional pelvic extraperitoneal radiotherapy, 3D-CRT and intensity-modulated radiotherapy developed in recent years can obtain the image information of lesions and adjacent normal tissues under the enhanced CT simulator and formulate the radiotherapy plan in combination with MRI, PET-CT, and other image diagnosis images [10]. Ali and others reported that during radiotherapy for cervical cancer, before cervical and uterine body displacement, the anterior and posterior directions of cervical and uterine body displacement are the largest [11]. Zhang and others performed imaging examination under different conditions on patients with radical cervical squamous cell carcinoma through multiple CT scans. The three-dimensional spatial coordinates of the reference center point in the CT image were compared with the bone reference point, and the influencing factors of the bladder skin on the positioning of target areas such as the cervix under different bladder skin filling degrees were analyzed. It was confirmed that the deviation of cervical lesions and uterine body in the *x*-axis direction was the smallest, and the mobility of cervical lesions and uterine body increased with the increase of bladder skin filling [12].

## 3. Experimental Analysis

### 3.1. Subjects

Patients with cervical cancer initially diagnosed as stage ia-iia2 and some stage III Cr (stage b1-iia2 of FIGO staging in 2009) from January 2018 to January 2019 were selected.

#### 3.1.1. Inclusion Criteria

1. Cervical cancer was diagnosed by pathological examination before operation. According to gynecological examination and imaging examination, the included cases were staged according to the FIGO staging standard in 2018
2. The initial treatment of all cases was radical hysterectomy + pelvic lymphadenectomy and abdominal paraaortic lymphadenectomy
3. All patients underwent whole abdominal enhanced CT scanning before operation
4. There was no preoperative infection and no other malignant tumor
5. Complete clinical and pathological data
6. This study obtained the consent of patients and their families and passed the review of the ethics committee of the hospital

#### 3.1.2. Exclusion Criteria

1. Preoperative radiotherapy or chemical therapy
2. Vaginal cancer and other primary tumors
3. Incomplete clinical or pathological data
4. The stage was late and there was no indication of operation

### 3.2. Research Methods

In this study, the new version of FIGO staging of uterine barium cancer in 2018 was used to revise the results of gynecological examination and imaging examination of cases of uterine barium cancer in Yili in 2018. IIICr patients included in the study were cervical cancer cases with the original clinical stage of I b1-II A2 [13, 14]. According to the size of lymph nodes measured by CT three-dimensional reconstruction technology, if the short diameter value is ≥10 mm, it is regarded as positive imaging lymph nodes, and the stage is IIICr stage. Because only a small number of cases have undergone abdominal paraaortic lymph node resection, IIIc stage in this study refers to the cases with positive pelvic lymph nodes. Then, according to the pathological results, whether lymph node metastasis is determined. If it is positive, it is defined as IIICp stage. In the process of clinical staging, two doctors above the level of deputy chief physician shall conduct gynecological examination to understand the general situation of cervical vagina and organs and tissues around the cervix, and then judge the focus and lymph node metastasis in combination with imaging examination to obtain the final staging.

The selection of diagnosis and treatment plan for patients with cervical cancer is based on FIGO staging and NCCN guidelines. Surgical treatment (radical hysterectomy + bilateral pelvic lymphadenectomy and abdominal paraaortic lymphadenectomy) is the main treatment. The operation shall be completed by doctors at or above the level of deputy chief physician. For stage IIICr, NCCN guidelines recommend concurrent radiotherapy and chemotherapy. However, since most of these patients are stage I A2-II A2 with or without lymph node metastasis according to the 2009 FIGO stage, most of the previous treatment will choose surgery. Therefore, for stage III C: patients with cervical cancer (stage I B1-II A2 in 2009 FIGO stage), surgery pathological staging (pelvic lymphadenectomy + paraaortic lymphadenectomy and sampling) can be performed before concurrent radiotherapy and chemotherapy [15].

#### 3.2.1. Data Import and Processing

The DICOM raw data obtained from CT scanning is directly imported into mimics 10.01 3D reconstruction software developed by Belgian materialise company to automatically complete image (tissue) positioning, obtain different cross-sectional data required for 3D reconstruction, and realize gray value insertion according to signal strength [16].

#### 3.2.2. Pelvic Lymph Nodes In Vivo

In two-dimensional CT images, pelvic lymph nodes usually show medium density circular or oval soft tissue shadow, which can be compared with surrounding fat. Anatomically, lymph nodes are mostly distributed along blood vessels and need to be distinguished from continuous arteriovenous. Import the obtained DICOM data of delay period into Mimics software; conduct operation through automatic positioning, interpolation processing, and other methods; and set the best reconstruction wide value (4-130 hu). After segmentation by using the threshold tool in the software editing tool (edit masks), draw the lymph nodes with the help of the sketching tool, and finally, calculate the reconstruction to obtain the corresponding three-dimensional model [17].

### 3.3. Statistical Methods

In this study, SPSS 18.0 software was used as the information processing tool. Measurement data should be presented as mean ± standard deviation and count data as frequency and percentage. For age as a continuous variable, the one-sample K-S test was used to test for normality; to compare ratios between groups, the chi-square test, univariate analysis, and Mann–Whitney *U* test were used to analyze differences in degree data. *P* < 0.05 indicates a statistically significant difference. Multivariate analysis ROC curves were drawn using logistic regression analysis, and the best predictors of blood SCC Ag and PLR were calculated. Using the results of lymph node analysis as the gold standard for evaluating lymph node metastasis, the sensitivity, specificity, positive predictive value, and negative predictive value of CT 3D reconstruction were calculated [18].

### 3.4. Result Analysis

204 patients with FIGO stage b1-II A2 in 2009 were selected. The diagnosis efficiency of MC stage was evaluated by CT three-dimensional reconstruction technology with the diagnosis of MCP as the gold standard. As shown in Table 1, 204 patients with cervical cancer underwent the construction of digital three-dimensional models of pelvic lymph nodes before treatment. It was found that 56 patients were diagnosed as stage III Cr; 60 cases of positive lymph nodes were found after operation, that is, 60 cases of stage III CP. At the same time, it is also concluded that with the increase of stage, the detection of lymph nodes by CT and pathology shows an upward trend [19].

The diagnostic effect of CT on lymph node metastasis in different clinical stages is further calculated as shown in Table 2. The CT diagnosis results of stage IIA lymph node metastasis are higher than those of stage IB, but the overall diagnostic accuracy of stage IIC is not high. The sensitivity and specificity were 52.86% and 80.56%, respectively, and the positive and negative predictive values were 56.92% and 77.85%, respectively. The results of IIICr and III CP stability studies showed that there was a correlation between CT and pathology in the diagnosis of lymph nodes, with a kappa value of 0.340. Insensitivity leads to an increased risk of misdiagnosis, i.e., stage III C indicates that a large proportion of postoperative disease is lymphadenopathy (IIICp), even if it was not diagnosed before surgery [20].

From January 2017 to January 2021, a total of 242 patients were diagnosed with cervical cancer for the first time in the Affiliated Hospital of the Third Medical University. Of these, 71 cases of pelvic lymphadenopathy were diagnosed as metastases in 29.3% (71/242). Their age distribution was 25-80 years [21], which was inconsistent with a normal distribution. As shown in Figure 2, the mean age was 50.86 ± 11.20 years, and the mean age was 51 years. The Mann–Whitney *U* test showed that there was no significant difference in age between patients with nonmetastatic lymph nodes and those with nonmetastatic lymph nodes (*P* = 0.139).

The age, FIGO stage, tumor diameter, tumor growth scheme, disease type, degree of differentiation, lymphatic invasion, interstitial invasion depth, uterine invasion, vaginal resection margin, and lymph node metastasis of 242 cervical cancer patients were statistically analyzed.  Table 3 shows that FIGO stage, tumor diameter, tumor growth protocol, disease type, degree of differentiation, lymphatic invasion, interstitial penetration depth, uterine cavity, and vaginal margin were statistically different between positive and negative lymph nodes. That is, pelvic lymph node metastasis is related to the above factors, and the *P* value is less than 0.05. Age was not associated with lymph node metastasis (*P* > 0.05).

Statistically significant risk factors examined by univariate analysis were analyzed using multivariate logistic regression methods. The results are shown in Table 4. Finally, differentiation, lymphatic invasion, depth of interstitial invasion, and uterine invasion were independent factors affecting lymph node metastasis (*P* < 0.05). Among them, parathyroid attack significantly affected lymph node metastasis (OR = 35.649, 95% confidence interval CI 4.356-291.739, *P* = 0.001); the incidence of pelvic lymph node metastasis was 5.806 times higher in patients with positive vascular invasion (OR = 5.806, 95% CI: 1.373-24.557; 0.017). The risk of lymph node metastasis was 3612 times higher in patients with incomplete cervical stromal invasion than in patients with invasive stroma < 1/2; 95% CI: 1.442-9.049; OR = 3.042, 95%, CI: 1.0-8.992. The greater the tissue difference, the lower the risk of pelvic lymph node metastasis [22, 23].

## 4. Discussion

The status of pelvic lymph nodes is closely related to the prognosis of cervical cancer and is an important factor in the choice of treatment for cervical cancer. The 2021nccn guidelines highlight node positivity as one of the risk factors for additional postoperative radiotherapy. Therefore, in clinical practice, it is clinically important to carefully evaluate whether cervical cancer patients develop pelvic metastases before treatment, that is, the following two conditions, mainly stage IIIC. First, imaging examination showed that lymph node enlargement was diagnosed as stage IIICr, but postoperative pathology confirmed that lymph nodes were negative, because not all enlarged lymph nodes in imaging examination were true metastasis. Because the latest guidelines did not recommend stratified treatment for stage III C patients, synchronous radiotherapy and chemotherapy were recommended for all these patients, which would make them miss the best time of surgical treatment and delay their condition; on the other hand, radiotherapy will make women of childbearing age lose ovarian function and thus lose reproductive function [24]. Second, imaging examination failed to find lymph node metastasis, but the operation showed positive lymph nodes (stage III CP). At this time, the patient needs to receive supplementary radiotherapy. This unnecessary lymph node dissection and radiotherapy will increase the total complications, such as lower limb lymphedema and pelvic lymph cyst with infection, and reduce the quality of life. Therefore, if we can judge whether lymph node metastasis is more accurate through imaging examination before treatment and improve the accuracy of stage III CX diagnosis, the prognosis of cervical cancer patients will be greatly improved.

At present, the conventional imaging methods used to predict cervical cancer lymph node metastasis include CT and MRI, which mainly rely on the short axis diameter of lymph nodes > lomm as the diagnostic standard. However, considering that cancer cell infiltration and reactive proliferation can lead to, the traditional imaging methods can not make accurate judgment, and their diagnostic value is medium. Therefore, some studies have confirmed that the size of lymph nodes combined with some imaging features, such as irregular shape or adhesion with surrounding tissues, ring enhancement after enhancement.

Cervical cancer is the second-largest female reproductive system malignancy after breast cancer. Patients with this disease account for 1/8 of all women with malignant tumors. Early determination of the condition of patients with cervical cancer and FIGO staging will help doctors to formulate an appropriate treatment plan as soon as possible and improve the effect of treatment. In the past, FIGO staging mainly depended on the subjective judgment of doctors, which required doctors to have solid theoretical knowledge and rich clinical experience. With the wide application of spiral CT in clinic, the results of multiphase enhanced spiral CT scanning and three-dimensional reconstruction technology have become an important basis for staging diagnosis of cervical cancer. The coincidence rate between the results of CT examination and pathological examination in these patients is high. When using spiral CT to examine patients with cervical cancer, the diameter of their lymph nodes can be measured on the cross-section, and then, the shape and location of lymph nodes can be reconstructed [25]. However, when this method is used to examine patients with cervical cancer, it has poor ability to distinguish the internal structure of lymph nodes and low sensitivity to lymph nodes with metastasis but small volume, especially lymph nodes with a diameter of less than 10 mm. This will make the diagnosis false positive or false negative. The detection rate and staging accuracy of these patients using spiral CT multiphase enhanced scanning and three-dimensional reconstruction technology are significantly higher than those using B-ultrasound. This is consistent with the results of relevant studies. It can be seen that the detection rate of cervical cancer diagnosed by spiral CT multiphase enhanced scanning and three-dimensional reconstruction technology is high, which is worthy of clinical application.

## 5. Conclusion

This study measured and analyzed the diameter of the three-dimensional model of pelvic lymph nodes. It was found that if the shortest diameter of lymph nodes ≥ 6.47 mm was used as the standard to judge the lymph node metastasis of cervical cancer, the diagnostic efficiency was improved, the sensitivity was 0.892, the specificity was 0.686, and the yoden index was 0.578. In order to make up for the deficiency of judging whether the lymph node is metastatic only by the short diameter value in clinical work, this study also combined the morphological standard of short length diameter ratio to comprehensively judge the metastatic lymph node. The normal lymph nodes without metastasis are long oval, and their short/long diameter ratio will be less than 0.5. The difference is that the abnormal positive lymph nodes tend to be spherical or irregular, and their short long diameter ratio is more than 0.5. With the help of digital three-dimensional reconstruction technology to reconstruct the three-dimensional model of pelvic lymph nodes, and accurately measure the relevant anatomical parameters, it is preliminarily concluded that taking the shortest diameter of lymph nodes ≥ 6.47 mm and the ratio of short to long diameter ≥ 0.57 as the diagnostic criteria, it has a certain reference value to judge lymph node metastasis.

This study selects the case study of our unit, which has selective bias on the selection of research objects. The small sample size has certain limitations on the research results. In this study, the diagnostic efficiency of three-dimensional reconstruction technology is moderate. The reason may be that the research department is retrospective study, the imaging equipment lacks advanced nature, and only the lymph node short diameter > l0 mm is the diagnostic standard. It cannot make correct judgment for normal size lymph nodes and lead to an increase in missed diagnosis rate. In addition, it is necessary to further combine other imaging features of lymph nodes, such as edge and enhancement, to improve the accuracy of diagnosis.

## Figures and Tables

**Figure 1:** 3D reconstruction technology.

**Figure 2:** Age distribution of patients.

**Table 1:** Determination of IIICr and IIICp in different clinical stages.

Clinical stages	Phase III C was determined by CT examination		Stage III C was determined by operation and pathology	
	Number of cases	Percentage	Number of cases	Percentage
IB (*n* = 158)	54	26.8%	46	28.7%
IIA (*n* = 56)	20	26.5%	21	40.1%
(*n* = 214)	56	29.4%	69	31.7%

**Table 2:** Diagnostic efficacy of CT in stage IIC at different clinical stages.

Clinical stages	Susceptibility	Specificity	Positive predictive value	Negative predictive value
IB	46.94%	7.08%	49.27%	78.95%
IIA	60.87%	75.83%	45.67%	74.29%
Total	52.87%	80.41%	73.92%	85.65%

**Table 3:** Variable test results for pelvic lymph node metastases in cervical cancer patients.

Clinicopathological factors	Negative lymph node metastasis	Positive lymph node metastasis	*X* ^2^/*z* value	*P* value
Age				
≤45	52	26	2.126	0.15
>45	118	35		
Stage				
IA	25	1	-5.740	<0.001
IB	78	19		
IIA	21	14		
IIICr	26	34		

**Table 4:** Multivariate logistic regression analysis of high-risk factors for lymph node metastasis.

Factor	Partial regression coefficient	Standard error	Wald	*P*	OR	95% CI
Degree of differentiation						
Low differentiation	—	—	10.952	0.004	—	—
Medium differentiation	-2.168	0.918	6.225	0.006	0.082	0.014-0.456
High differentiation	-2.280	1.029	11.842	0.001	0.043	0.005-0.254

## Data Availability

The data used to support the findings of this study are available from the corresponding author upon request.
